This article has been retracted.

# Efficacy and Prediction Model Construction of Drug-Coated Balloon Combined with Cutting Balloon Angioplasty in the Treatment of Drug-Eluting Stent In-Stent Restenosis

**DOI:** 10.1155/2022/9832622

**Published:** 2022-09-19

**Authors:** Haokun Wu, Tianhao Yu, Ting Fan, Wenjun Liao

**Affiliations:** Guangdong Second Provincial General Hospital, Guangzhou, Guangdong 510317, China

## Abstract

**Objective:**

To investigate the efficacy of drug-coated balloon (DCB) combined with cutting balloon angioplasty (CBA) in the treatment of drug-eluting stent in-stent restenosis (DES-ISR) and to construct a predictive model for the occurrence of DES-ISR.

**Methods:**

According to the criteria of diagnosis, inclusion, and exclusion, DES-ISR patients who were treated in the outpatient and inpatient departments of cardiovascular medicine of Second People's Hospital of Guangdong Province from July 2021 to December 2021 were included. A total of 72 cases were planned to be enrolled, including 36 cases in the control group and 36 cases in the experimental group. The control group was treated with DCB, and the experimental group was combined with CBA. The treatment success rate, coronary angiography results before and after surgery, and the incidence of major adverse cardiovascular events during the follow-up period were compared between the two groups. Seventy-two DES-ISR patients were divided into ISR group and 59 non-ISR patients were divided into non-ISR group. The clinical data of the two groups were compared to analyze the risk factors affecting the occurrence of DES-ISR, and the prediction model was established.

**Results:**

The surgical success rate of the experimental group was 94.44% (34/36), which was higher than the 77.78% (28/36) of the control group (*P* < 0.05). The minimum lumen diameter (MLD) of the experimental group 6 months after operation was greater than that of the control group, the late lumen loss (LL) and lumen stenosis rate were higher than those in the control group, and the incidence of major adverse cardiovascular events was lower than that in the control group (*P* < 0.05). In the ISR group, the proportion of patients with abnormal BMI, smoking, hypertension, diabetes, and family history of coronary heart disease and multivessel coronary artery disease was higher than that in the non-ISR group, the degree of stenosis target lesion was higher than that in the non-ISR group, the diameter of target lesion and stent diameter were smaller than those in the non-ISR group, and the length of target lesion and stent length were longer than those in the non-ISR group; the number of stents was more than that in the non-ISR group (*P* < 0.05). Combined hypertension, multiple coronary artery lesions, stenosis target lesion degree ≥85.05%, and target lesion length ≥36.88 mm were risk factors for DES-ISR, and target lesion diameter ≥3.15 mm and stent diameter ≥3.15 mm were protective factors (*P* < 0.05). The prediction model of DES-ISR was obtained by multiple logistic regression analysis, *P* = 1[1 + *e*^(2.281 + 3.321X_hypertension_ + 3.427X_umber of arterial lesions_ + 3.359X_stenosis target lesion degree_ − 3.143X_target lesion diameter_ + 0.650X_target lesion length_ − 10.159X_stent diameter_)^]. The Hosmer-Lemeshow test showed that Hosmer-Lemeshow *χ*^2^ = 0.925, *P* =0.413; the ROC curve analysis showed that the AUC of the prediction model for the occurrence of DES-ISR was 0.924, the SE value was 0.022, and the 95% CI was 0.880-0.967.

**Conclusion:**

DCB combined with CBA has good clinical efficacy in the treatment of DES-ISR, which can reduce the rate of lumen stenosis and the incidence of adverse cardiovascular events. The prediction model established according to risk factors has high predictive value for the occurrence of DES-ISR.

## 1. Introduction

Coronary atherosclerotic heart disease is a heart disease caused by atherosclerotic lesions in the coronary vessels, resulting in stenosis or obstruction of the vascular lumen, resulting in myocardial ischemia, hypoxia, or necrosis [1]. At present, 7.3 million people die of ischemic heart disease every year in the world, ranking first among all diseases, accounting for 12.8% of all deaths from diseases [2]. Currently, percutaneous coronary drug-eluting stent (DES) has become the main means for the treatment of coronary heart disease, but the occurrence of in-stent restenosis (ISR) limits its long-term clinical benefits [3]. Although DES has been widely used and the design of stent structures has been continuously improved, the incidence of ISR in patients with DES is still as high as 10% [4]. ISR refers to restenosis of coronary artery in-stent lesions caused by coronary artery endothelial injury and gradual proliferation of intimal tissue caused by percutaneous coronary interventional therapy, and its mechanism includes biological, mechanical, and technical factors [5]. Relevant studies have pointed out that due to factors such as poor vascular endothelialization, local allergic reactions, and individual differences, there are still a considerable proportion of patients with adverse clinical and anatomical characteristics, and the analysis of risk factors affecting the occurrence of ISR in patients and effective intervention can reduce the risk of ISR [6, 7]. Balloon dilation is the main treatment for ISR. Domestic studies have shown that, compared with conventional high-pressure balloons, cutting balloon angioplasty (CBA) can squeeze and cut plaques to a certain extent, reduce complications such as vascular dissection and loss, and can increase immediate lumen acquisition rate and minimum lumen area after stent implantation [8]. Previous studies have pointed out that because of its ability to provide anti-restenosis drugs to the vascular endothelium and the avoidance of multilayer stent implantation, the drug-coated balloon (DCB) has received different clinical indications including the treatment of ISR in the past few years [9]. Therefore, this study combined the two in the clinical treatment of DES-ISR, aiming to explore its clinical efficacy on DES-ISR, and to construct a prediction model for the occurrence of DES-ISR, so as to provide reference for the clinical prevention and treatment of the disease.

## 2. Materials and Methods

### 2.1. Clinical Data

DES-ISR patients treated in the outpatient and inpatient departments of Department of Cardiovascular Medicine of the Second People's Hospital of Guangdong Province from July 2021 to December 2021 were included according to diagnosis, inclusion, and exclusion criteria. A total of 72 cases were planned to be enrolled, including 36 cases in the control group and 36 cases in the experimental group. There was no significant difference in general data between the two groups (*P* > 0.05), as shown in Table 1. This study has been approved by the hospital medical ethics committee.

#### 2.1.1. Diagnostic Criteria

ISR is diagnosed according to relevant guidelines [10]: multi-projection coronary angiography or intracoronary imaging examinations indicated that the diameter of the stent lumen of the coronary target vessel has a stenosis of ≥50%, including coronary artery within 5 mm of both ends of the stent.

#### 2.1.2. Inclusion Criteria

(1) Aged 18-80 years old, male or non-pregnant woman; (2) patients treated with DCB implantation and diagnosed with ISR 6-12 months after operation; (3) lesion length ≤40 mm; (4) subjects who understood the purpose of the experiment, voluntarily participated, and signed the written informed consent; (5) patients diagnosed with DES-ISR by coronary angiography after 6-9 months of PCI; (6) complete clinical data.

#### 2.1.3. Exclusion Criteria

(1) Patients allergic to paclitaxel drugs; (2) patients with contraindications of antithrombotic drugs; (3) patients who were intolerant or allergic to more than one anti-platelet aggregation drug; (4) patients with myocardial infarction within one week; (5) patients with history of cerebrovascular accident or peptic ulcer or gastric bleeding within 6 months, or who were judged to be bleeding constitution by researchers; (6) restenosis in left main trunk stent; (7) lesion length >40 mm; (8) there was more than one layer of stent in the target vessel; (9) ISR lesions with residual stenosis >40% after conventional pretreatment; (10) glycated hemoglobin ≥9%; (11) patients with other types of heart disease; (12) subjects had poor compliance and could not complete the study as required.

#### 2.1.4. Criteria for Dropout and Exclusion of Cases

(1) Those who did not meet the criteria and were mistakenly included; (2) patients who failed to follow the prescribed treatment regimen after inclusion; (3) patients whose treatment was discontinued or lost to follow-up for other reasons resulting in missing or no test records. For the included cases, those who meet one of the above criteria were excluded. All the excluded cases should be explained the reasons for exclusion, and their observation table should be kept for future reference

### 2.2. Methods

#### 2.2.1. Control Group

The target blood vessel was examined by IVUS, and the high-pressure balloon was fully predilated. DCB of appropriate size was selected after coronary angiography showed no dissection, residual stenosis of less than 40%, and distal blood flow of TIMI grade 3 (Yinyi Biological Technology Co., LTD, Qingzhou® Coronary Drug Delivery System). The relevant longitudinal length of its expanded area should be larger than that of the pre-expanded balloon, and the diameter of DCB should be higher than that of the pre-expanded balloon, so as to ensure that DCB can cover the pre-expanded area by 2-3 mm on both sides and prevent the geographical loss of DCB. The operation should be carried out as soon as possible after the DCB contacted the blood, and the expansion time was 60-90s. IVUS examination was performed after treatment.

#### 2.2.2. Treatment Method of Experimental Group

IVUS was used to examine the target vessels, and the high-pressure balloon was fully predilated, and then a cutting balloon was used to dilate the lesions (the model of the cutting balloon was selected according to the ratio of 1 : 1 to the actual stent diameter). During the dilation of the lesion, the cut balloon was slowly pressurized and predilated for 2 to 3 times. DCB was applied and other steps were the same as the control group after coronary angiography showed no dissection, residual stenosis of less than 40%, and distal blood flow of TIMI grade 3.

### 2.3. Clinical Data Collection

The patient's baseline data and clinical data were collected using the information system of hospital, mainly including demographic characteristics [age, gender, BMI (normally 18.5 ~ 23.9 kg/m^2^), etc.], cardiovascular risk factors (such as smoking, hypertension, diabetes, hypercholesterolemia, hyperuricemia, and family history of coronary heart disease), angiographic information (such as multivessel disease, target lesion location, double vessel disease, degree of stenosis target lesion, and length of target lesion), surgical steps (such as stent length and stent diameter), and postoperative medication (such as statins, beta-blockers, ACEIs, ARBs, and calcium channel blockers).

### 2.4. Evaluation Criteria of Curative Effect [11]

Successful treatment: after treatment, the lumen of the target vessels was significantly enlarged, the residual stenosis of the main branch vessels was <20%, and the residual stenosis of the branch vessels was <30%. Angiography showed that blood flow of TIMI grade 3 was obtained, and there were no major clinical complications during hospitalization, and no recurrence occurred 6 months after surgery.

### 2.5. Coronary Angiography

All patients underwent coronary angiography before surgery, immediately after surgery, and 6 months after surgery. Coronary quantitative analysis software was used to analyze the imaging data of coronary angiography, mainly including minimal lumen diameter (MLD), reference vessel diameter (RVD), late lumen loss (LL), and lumen stenosis rate.

### 2.6. Statistical Processing

SPSS 22.0 software was used to process data, enumeration data were expressed as %, and differences between groups were compared by *χ*^2^ test; measurement data were expressed as ^−^*x* ± *s* after normality test, and differences between groups were compared by *t* test. Logistic regression was used to analyze the risk factors for DES-ISR. The Hosmer-Lemeshow test was used to analyze the degree of fitting between the prediction model and the standard curve. ROC curve was used to analyze the predictive value of the model for DES-ISR occurrence. *P* < 0.05 indicated that the difference was statistically significant.

## 3. Results

### 3.1. Comparison of Therapeutic Effects between the Two Groups

The surgical success rate of the experimental group was 94.44% (34/36), which was higher than 77.78% (28/36) of the control group (*χ*^2^ = 0.041, *P* < 0.05).

### 3.2. Comparison of Coronary Angiography Results between the Two Groups before and 6 Months after Surgery

There was no significant difference in preoperative RVD and MLD immediately after operation between the two groups (*P* > 0.05); the MLD of the experimental group was higher than that of the control group 6 months after surgery, and the LL and lumen stenosis rate were higher than those of the control group (*P* < 0.05), as shown in Table 2.

### 3.3. Comparison of the Incidence of Major Adverse Cardiovascular Events between the Two Groups

The incidence of major adverse cardiovascular events in the experimental group was lower than that in the control group (*P* < 0.05), as shown in Table 3.

### 3.4. Univariate Analysis of Factors Affecting the Occurrence of DES-ISR

In the ISR group, the proportion of patients with abnormal BMI, smoking, hypertension, diabetes, and family history of coronary heart disease and multivessel coronary artery disease was higher than that in the non-ISR group, the degree of stenosis target lesion was higher than that in the non-ISR group, the diameter of target lesion and stent diameter were smaller than that in the non-ISR group, the length of target lesion and stent was longer than that in the non-ISR group, and the number of stents was higher than that of the non-ISR group (*P* < 0.05), as shown in Table 4.

### 3.5. Multivariate Analysis of Factors Affecting the Occurrence of DES-ISR

Combined hypertension, multivessel coronary lesions, stenosis target lesion degree ≥85.05%, and target lesion length ≥36.88 mm were risk factors affecting the occurrence of DES-ISR, and target lesion diameter ≥3.15 mm and stent diameter ≥3.15 mm were protective factors (*P* < 0.05), as shown in Table 5.

### 3.6. Establishment of the Prediction Model and Analysis of the Calibration Degree of the Model

The prediction model of the occurrence of DES-ISR was obtained by multivariate logistic regression analysis, *P* = 1[1 + *e*^(2.281 + 3.321X_hypertension_ + 3.427X_number of arterial lesions_ + 3.359X_stenosis target lesion degree_3.143X_target lesion diameter_ + 0.650X_target lesion length_ − 10.159X_stent diameter_)^]. The Hosmer-Lemeshow test showed that Hosmer-Lemeshow *χ*^2^ = 0.925, *P* =0.413, as shown in Figure 1.

### 3.7. Prediction Efficiency Analysis of the Prediction Model

According to the ROC curve analysis, the AUC of the prediction model to predict the occurrence of DES-ISR was 0.924, the SE value was 0.022, and the 95% CI was 0.880-0.967, as shown in Figure 2.

## 4. Discussion

ISR is a major clinical problem after interventional therapy, which is mainly caused by coronary intimal hyperplasia, and oral administration alone to reduce the incidence of ISR is ineffective and has side effects [12]. Relevant studies have pointed out that DCB treatment for DES-ISR patients can improve the degree of in-stent stenosis [13, 14]. It has also been reported that CBA can reduce the incidence of repeated ISR and have less lumen loss than ordinary high-pressure balloon preconditioning [15, 16]. DCB is a commonly used treatment for coronary artery diseases, which can treat stenosis or occlusive vascular diseases by carrying chemotherapy drugs to the surface of the diseased vessels. The chemical drug paclitaxel on its surface makes full contact with the vascular wall of the lesion through balloon dilation and quickly penetrates into the arterial wall to inhibit intimal hyperplasia and prevent vascular restenosis [17, 18]. Studies have shown that although DCB can release anti-proliferative drugs to the coronary vascular wall through balloon dilation of local vessels to achieve the effect of inhibiting intima hyperplasia, some patients will still have adverse cardiovascular events in later stage, which affects the prognosis [19, 20]. Some scholars have found that the combination of CBA on the basis of DCB in the treatment of ISR can achieve a better therapeutic effect [21, 22]. This study found that the surgical success rate of the experimental group was higher than that of the control group, and after 6 months of surgery, the MLD, LL, and the lumen stenosis rate were higher than those of the control group, indicating that DCB combined with CBA has a good clinical effect on the treatment of DES-ISR and can reduce the lumen stenosis rate. The reason is that the drug balloon effectively reduces the inflammatory response of the intima of blood vessels and inhibits intima hyperplasia in the short term after surgery. In addition, precise expansion with CBA can prevent the balloon from sliding out of the stent, resulting in stent edge injury. Cutting treatment can cut the new intima tissue, which is theoretically helpful for the uptake of drugs delivered by DCB, thus improving the therapeutic effect [23]. In addition, the results show that combined treatment can reduce the incidence of adverse cardiovascular events, which is mainly related to the fact that CBA can squeeze and cut plaque to a certain extent, reduce complications such as vascular dissection and loss, and increase the immediate lumen acquisition rate, and retreatment reduces the circumferential force of the blood vessel wall and reduces the elastic recoil rate of the blood vessel wall [24].

Clinical data showed that the occurrence of DES-ISR was mainly related to local factors such as stent margins and the focal site, and it mostly occurred 6 months after surgery [25, 26]. It has been reported that the causes of ISR mainly include insufficient stent expansion, abnormal intimal hyperplasia, or new atherosclerosis, but the risk factors for the occurrence of DES-ISR are still inconclusive [27]. Therefore, this study analyzed the relevant factors affecting its occurrence. Related reports have shown that after coronary stenting, there is a significant correlation between diabetes and ISR, and diabetes is associated with clinical outcomes such as stent thrombosis and major adverse cardiac events after PCI [6]. ISR may occur in diabetic patients due to insulin resistance and complex underlying lesions. However, the results of this study showed that it was not related to the occurrence of ISR, which may be related to the small sample size of this study, so the sample size should be increased for further analysis in the later stage. Previous studies have found that the characteristics of coronary artery lesions, including the number of vessels, length, location, nature, and stenosis degree of coronary artery lesions, can affect the occurrence of ISR [28]. Studies have confirmed that the incidence of ISR in patients with multivessel lesions is higher than that in patients with single-vessel lesion. The diameter of diseased vessels and the length of total lesions are also predictors of restenosis, and the incidence of ISR increases significantly when the diameter of vessels is too small [29] .In this study, it was found that multivessel coronary artery lesions, stenosis target lesion degree ≥85.05%, and target lesion length ≥36.88 mm were risk factors affecting the occurrence of DES-ISR, and target lesion diameter ≥3.15 mm and stent diameter ≥3.15 mm were protective factors. It indicates that the increased length of implanted stents and the smaller diameter of stents significantly increase the incidence of ISR. The matching of the stent diameter and the diameter of the blood vessel is very important to reduce the risk of restenosis, and longer stents are important risk factors for restenosis and ST. This study also found that hypertension is also a risk factor for the occurrence of ISR, which is mainly related to vascular endothelial dysfunction in patients with hypertension.

At present, it is believed that identifying possible high-risk patients with ISR through the predictive model will help clinicians to carry out targeted doctor-patient communication and health education, so that patients can clearly realize the importance of postoperative rehabilitation. Adhering to the secondary prevention of coronary heart disease and developing individualized control programs for high-risk factors can theoretically further reduce the incidence of ISR after PCI, thus improving the expected prognosis of patients as much as possible. In this study, a prediction model was established according to various risk factors. The Hosmer-Lemeshow test and ROC curve analysis showed that the model has high predictive value for the occurrence of ISR, so it may be applied to the early prediction of ISR.

In conclusion, DCB combined with CBA has good clinical efficacy in the treatment of DES-ISR, which can reduce the rate of lumen stenosis and the incidence of adverse cardiovascular events. The prediction model established according to risk factors has high predictive value for the occurrence of DES-ISR in patients.

## Figures and Tables

**Figure 1:** Calibration analysis of the prediction model.

**Figure 2:** ROC curve analysis of the prediction model predicting the occurrence of DES-ISR.

**Table 1:** Comparison of general data between the experimental group and the control group.

General data	Experimental group (*n* =36)	Control group (*n* =36)	*χ* ^2^/*t*	*P*
Gender male (cases)	20	22	0.229	0.633
Age (years)	67.28 ± 5.04	66.06 ± 5.01	1.030	0.307
Abnormal BMI (cases)	20	23	0.520	0.471
Smoking (cases)	17	18	0.056	0.814
Hypertension (cases)	14	17	0.510	0.475
Diabetes (cases)	15	17	0.225	0.635
Hyperlipidemia (cases)	4	6	0.465	0.496
Family history of coronary heart disease (cases)	18	17	0.056	0.814

**Table 2:** Comparison of coronary angiography results between the two groups before and 6 months after surgery.

Group	*n*	MLD (mm)		Lumen stenosis rate (%)		RVD (mm)	LL (mm)
		Immediately after surgery	Six months after surgery	Before surgery	Six months after surgery		
Experimental group	36	0.98 ± 0.17	1.79 ± 0.32	69.78 ± 5.31	24.19 ± 3.19	2.89 ± 0.47	0.51 ± 0.13
Control group	36	0.96 ± 0.19	1.51 ± 0.28	71.57 ± 5.05	30.07 ± 3.52	2.83 ± 0.51	0.67 ± 0.14
*t*		0.471	3.951	1.466	7.427	0.519	5.025
*P*		0.639	<0.001	0.147	<0.001	0.605	<0.001

**Table 3:** Comparison of the incidence of major adverse cardiovascular events between the two groups (cases, %).

Group	*n*	Target vessel revascularization	Target lesion revascularization	Nonfatal myocardial infarction	All-cause mortality	Incidence
Experimental group	36	1	0	2	1	11.11 (4)
Control group	36	2	1	5	2	30.56 (11)
*χ* ^2^						4.126
*P*						0.042

**Table 4:** Univariate analysis of factors affecting the occurrence of DES-ISR.

Factors	ISR group (*n* =72)	Non-ISR group (*n* =59)	*χ* ^2^/*t* value	*P* value
Age (years)	65.08 ± 5.38	64.34 ± 5.07	0.804	0.423
Gender (cases)				
Male	42	35	0.013	0.909
Female	30	24		
Abnormal BMI (cases)	43	20	8.663	0.003
Smoking (cases)	35	13	9.866	0.002
Hypertension (cases)	31	9	11.816	0.001
Diabetes (cases)	32	11	9.789	0.002
Hyperlipidemia (cases)	10	8	0.003	0.957
Family history of coronary heart disease (cases)	35	12	11.267	0.001
Platelets (∗10^11^)	1.07 ± 0.19	1.13 ± 0.24	1.597	0.113
LVEF (%)	60.32 ± 5.09	59.83 ± 5.11	0.547	0.585
Number of arterial lesions (cases)				
Multivessel lesions	61	29	19.081	<0.001
Single-vessel lesion	11	30		
Target lesion location (cases)				
Anterior descending branch	42	34	0.009	0.996
Circumflex branch	13	11		
Right coronary artery	17	14		
Stenosis target lesion degree (%)	88.34 ± 3.16	81.62 ± 3.86	10.958	<0.001
Target lesion diameter (mm)	2.85 ± 0.51	3.51 ± 0.59	6.866	<0.001
Target lesion length (mm)	41.69 ± 4.32	31.53 ± 5.04	12.422	<0.001
Stent implantation time (years)	4.07 ± 0.59	4.13 ± 0.67	0.545	0.587
Stent length (mm)	23.58 ± 2.73	21.09 ± 2.25	5.614	<0.001
Stent diameter (mm)	3.09 ± 0.18	3.26 ± 0.16	5.651	<0.001
Number of stents	1.95 ± 0.32	1.53 ± 0.21	8.665	<0.001
Postoperative medication (cases)				
Statins	71	56	0.862	0.930
Beta-blockers	59	48		
ACEI	37	34		
ARB	18	11		
Calcium channel blockers	30	25		

**Table 5:** Multivariate analysis of factors affecting the occurrence of DES-ISR.

Index	*β*	*SE*	Wald's *χ*^2^	*OR*	*95% CI*	*P* value
Abnormal BMI	2.281	1.282	3.166	9.786	0.793~120.750	0.076
Smoking	2.153	1.328	2.628	8.611	0.638~116.266	0.106
Hypertension	3.321	1.501	4.895	27.688	1.461~524.770	0.027
Diabetes	0.248	1.196	0.043	1.281	0.123~13.359	0.836
Family history of coronary heart disease	2.487	1.273	3.817	12.025	0.992~145.777	0.051
Number of arterial lesions	3.427	1.458	5.525	30.784	1.767~536.293	0.019
Stenosis target lesion degree	3.359	1.298	6.697	28.760	2.259~366.164	0.010
Target lesion diameter	-3.143	1.355	5.380	0.043	0.003~0.614	0.021
Target lesion length	0.650	0.211	9.490	1.916	1.267~2.897	0.002
Stent length	2.798	1.434	3.807	16.412	0.987~272.773	0.052
Stent diameter	-10.159	3.452	8.661	0.000	0.000~0.034	0.003
Number of stents	0.099	1.112	0.008	1.104	0.125~9.762	0.929
Constant	2.281	1.282	3.166	9.786	0.793~120.750	0.076

Assignment: abnormal BMI (yes was 1, no was 0); smoking (yes was 1, no was 0); hypertension (yes was 1, no was 0); diabetes (yes was 1, no was 0); family history of coronary heart disease (yes was 1, no was 0); number of coronary artery lesions (multiple vessels was 1, single vessel was 0); stenosis target lesion degree (≥85.05% was 1, <85.05% was 0); target lesion diameter (≥3.15 mm was 1, <3.15 mm was 0); stent diameter (≥3.15 mm was 1, <3.15 mm was 0); target lesion length (≥36.8 mm was 1, <36.88 mm was 0); stent length (≥22.07 mm was 1, <22.07 mm was 0); number of stents (≥2 was 1, <2 was 0).

## Data Availability

The labeled dataset used to support the findings of this study is available from the corresponding author upon request.
